The article "Comprehensive Health Evaluation Model of Art Psychotherapy Using Genetic Algorithm" was retracted in 2023. Reasons: unreliable results or conclusions; concerns about the data; concerns about the results or conclusions; concerns about the peer review.

# Comprehensive Health Evaluation Model of Art Psychotherapy Using Genetic Algorithm

**DOI:** 10.1155/2022/5718050

**Published:** 2022-08-02

**Authors:** Fupeng Zhang, Xia Liu

**Affiliations:** ^1^Luliang University, Luliang 033001, China; ^2^Jeonju University, Jeonju-si 55068, Republic of Korea

## Abstract

In order to explore the real effect of art mental health therapy, this paper proposes a feature selection algorithm based on genetic algorithm. The algorithm takes college students as the research object and discusses the effect of psychotherapy on college students through painting art therapy. The results showed that there were extremely significant differences in EPQ extraversion factors among the people treated with the educational intervention of art psychology course (*P* < 0.01), and there was no significant change in other factors (*P* > 0.05). There was no significant change in total depression score and depression index (*P* > 0.05). There were significant differences in social avoidance factors and social anxiety (*P* < 0.05), and there were relatively significant differences in the total score of sadness (*P* < 0.01). It is concluded that the use of artistic elements can effectively help people express themselves and express their psychological emotions, which has a certain effect in mental health treatment.

## 1. Introduction

Before the formation of language and words, early human beings mainly used graphics and painting to record events in life and through graphics to reflect emotions and ideas of colossus. Therefore, the artistic expression in the form of graphics and painting is the innate instinct of human beings. The key point of artistic therapy is to effectively integrate different forms of art types into psychotherapy and, at the same time, use artistic media such as painting, music, and dance to promote the growth of people's mind and cure people's psychological problems in a supportive environment. Therefore, art psychotherapy is also a process of discovering and expressing oneself with the help of art forms derived from the depths of emotion. And in the process of self-psychotherapy using art forms, people usually do not pay too much attention to the beauty of visual art, the grammatical arrangement of words, and the harmony and fluency of songs. They just use art to release, express and relax, and obtain insight by studying symbolic and metaphorical information to achieve the effect of psychotherapy, as shown in Figure 1.

## 2. Literature Review

Modern psychotherapy with speech as the medium has a good effect in correcting irrational cognition and thinking, but it is powerless in dealing with psychological problems with emotional distress as the main symptoms, such as emotional disorder and traumatic experience. In brain science, emotion and art (painting, music, etc.) are controlled by the right hemisphere at the same time. Therefore, even speech therapists with rich clinical experience do not despise the excellent effect of painting in dealing with emotional distress. A large number of studies abroad have proved the artistic way of using the right hemisphere to deal with emotional disorder [1].

The article "Comprehensive Health Evaluation Model of Art Psychotherapy Using Genetic Algorithm" was retracted in 2023. Reasons: unreliable results or conclusions; concerns about the data; concerns about the results or conclusions; concerns about the peer review.

Children with family and development problems were treated with spontaneous painting creation method. It was found that painting therapy can alleviate the pressure from family and society, express anxiety, and strengthen the self-concept of visitors [2]. Individual and group painting therapy was carried out for children with learning disabilities. It was found that, in the treatment, children and peers promoted the development of social skills through interpersonal interaction and finally improved individual self-esteem. Babin applied painting psychotherapy to 3 women with anorexia and 3 women with obesity. The results showed that the self-concept of 5 women was significantly improved [3]. It is found that painting intervention can promote homeless women to improve their sense of self-esteem and self-awareness. The research of some scholars has found a physiological basis for painting to promote the improvement of self-esteem. He found that fluctuations in the amount of neurotransmitter serotonin in the brain can affect the quality of movement and the level of self-esteem. The high content of serotonin is related to self-affirmation and movement control, and the low content is easy to lead to anger and impulsive behavior. Human life depends on movement, and effective and elegant movement produces a sense of satisfaction. The training provided by art happens to produce such skill movements. The display of these movements leads to positive feedback among people, thus strengthening self-esteem [4].

Since the 1940s, psychologists have also developed a variety of painting projection techniques for psychotherapy and testing, but basically painting projection techniques can be divided into three categories: free painting, painting with specified content, and painting techniques in between. The first is free painting technology. The stimulation given is only paper and pen, giving the visitor the greatest freedom to express the inner world he is most eager to express. However, analysts need extensive knowledge background and rich analysis experience, which makes it difficult to quantify and ensure reliability and validity. The second category is the painting technology that specifies the content. Fang Shuren painting test is the most comprehensive and widely used typical representative. It gives standard guidelines and has certain provisions on content, tools, and location, which is more conducive to the popularization of experience and application in experimental research. The last one is between the two. It gives a certain stimulation, but it does not regulate what content to paint at the same time. In addition, the final analysis of this technology is not for the painting content of the subjects, but for the nature of the changes made by the subjects on the given stimulus [5].

The article "Comprehensive Health Evaluation Model of Art Psychotherapy Using Genetic Algorithm" was retracted in 2023. Reasons: unreliable results or conclusions; concerns about the data; concerns about the results or conclusions; concerns about the peer review.

Domestic painting psychotherapy has also achieved some applied research results in the treatment and diagnosis of mental disorders, special groups such as intellectual disabilities, crisis intervention and psychological education, and group psychological counseling and treatment [6].

In the study of a case of children's depression, painting image was used to regulate children's depression, and the effect was remarkable. This paper discusses the application of painting therapy in middle school students with emotional disorders and uses the room tree person test method to treat 6 middle school students who come to psychological counseling. It is found that the use of painting therapy can better understand the causes of middle school students' emotional conflict and has played a good effect in the process of psychological counseling. The study tried to use painting projection technology, free association, and positive imagination in a psychological counseling case of depression to fully present the patient's past experience, internal image, and unconsciousness and communicate the patient's consciousness and unconsciousness. The results show the patient's inner growth and development, and the performance has been changed and transformed in real life. Through the experimental treatment of college students' depressive symptoms through painting aesthetic treatment activities, the results show that the design can significantly improve the level of college students' depressive symptoms, promote the college students with depressive symptoms, and significantly improve the overall mental health level of the subjects. Its effect is mainly reflected in the significant improvement of four factors: somatization, interpersonal sensitivity, psychosis, and paranoia [7].

A team explored the effect of group painting art therapy on the rehabilitation of physiological, psychological, and social functions of schizophrenic patients. The results show that group painting art intervention can alleviate the mental symptoms of schizophrenic patients and promote the improvement of patients' self-concept and quality of life. The application of painting therapy in interpersonal group counseling is an effective method for college students with development crisis, personality problems, and international communication problems. Through group counseling, the self-acceptance of members can be improved, the sense of self-harmony can be enhanced, and the level of self-esteem can be improved to varying degrees. Group counseling promotes the personality growth of members as a whole and improves their mental health level. Collective painting therapy starts from the two points of collectivity and painting to easily create a treatment environment and guide most people. Patients talked about its novelty and being easy to understand after treatment. As an auxiliary form of psychotherapy, painting therapy has its uniqueness [8].

The article "Comprehensive Health Evaluation Model of Art Psychotherapy Using Genetic Algorithm" was retracted in 2023. Reasons: unreliable results or conclusions; concerns about the data; concerns about the results or conclusions; concerns about the peer review.

## 3. Unsupervised Feature Selection Algorithm Based on Genetic Algorithm

### 3.1. Feature Selection Algorithm

Feature selection, at first, is a technology in the classification problem. The purpose is to find out which features have a great influence on the label, minimize the influence of irrelevant features in the classifier training process, and avoid overfitting and high time complexity. From the definition, the process of feature engineering is mainly composed of the following aspects, as shown in Figure 2.

Feature selection algorithms often use some evaluation criteria to measure the candidate subsets. The evaluation criteria are divided into two categories according to whether they are related to the subsequent machine learning model. One kind of evaluation criteria is independent of the learning model and evaluates the feature selection as an independent process. This feature selection algorithm is called filter algorithm. This feature selection process is shown in Figure 3 below.

The other is called wrapper algorithm. In this algorithm, the evaluation criterion is the performance of the subsequent machine learning model. In this process of machine learning, feature selection is a part of the establishment of machine learning model [9]. For each candidate feature subset, the model needs to be retrained. The specific process is shown in Figure 4.

In the field of practical application, when the feature dimension is high and there are many redundant features, these two hybrid strategies are often used for feature selection. Firstly, the independent evaluation criterion algorithm is used to preliminarily evaluate the features and quickly eliminate most irrelevant features. Then, the encapsulated feature selection is carried out for the remaining few features to obtain the feature subset with the best neutral energy for the subsequent machine learning model [10].

The article "Comprehensive Health Evaluation Model of Art Psychotherapy Using Genetic Algorithm" was retracted in 2023. Reasons: unreliable results or conclusions; concerns about the data; concerns about the results or conclusions; concerns about the peer review.

### 3.2. Genetic Algorithm

#### 3.2.1. Conceptual Process

The core idea of the algorithm is to characterize the iterative process of the solution of the optimization problem by the heredity of genes in the population. Among them, the population represents the set of all feasible solutions, and each individual gene in the population represents a feasible solution. By artificially setting a natural environment (fitness function, or evaluation function), the way of survival of the fittest in nature is simulated. Filter the individuals in the population that are not suitable for the natural environment and inherit the individual genes suitable for the environment. Through the characteristics of gene crossover and variation in the genetic process, the offspring population can not only retain the characteristics of good solutions in the previous generation population, but also retain the possibility of producing better solutions [11]. The flow of genetic algorithm is shown in Figure 5 below.

In the feature selection problem, as shown in Figure 6, for a data set with feature number *n*, a binary gene sequence with length *n* is usually used to represent a feasible solution. In each gene, 0 indicates that the feature is not in the individual, and 1 indicates that the feature exists in the individual. Each coding sequence represents an individual [12].

#### 3.2.2. Definition of Population Genetic Mode

Roulette selection algorithm: roulette selection algorithm comes from roulette gambling. The main principle is that, on the roulette surface, regions with different angles have different probability of being selected; that is, the larger the proportion, the easier it is to be selected. In the feature selection algorithm, the higher the fitness, the easier it is to be selected. In a population with *N* individuals, for individual *x*_*i*_, given its fitness *f*(*x*_*i*_), the probability of individual selection is carried out according to the following algorithm:

(1) Use formula (1) below to calculate the individual fitness ratio, which is similar to the ratio of different areas on the roulette.
  (1) $$\begin{array}{c} p\left(x_{i}\right)=\frac{f\left(x_{i}\right)}{\sum_{j=1}^{N}f\left(x_{i}\right)}. \end{array}$$
(2) Calculate the cumulative fitness distribution from *x*_1_ to *x*_*N*_, similar to the probability distribution function, as shown in formula (2) below:
  (2) $$\begin{array}{c} q_{i}=\sum_{j=1}^{i}p\left(x_{i}\right). \end{array}$$
(3) Take random number as shown in formula (3):
  (3) $$\begin{array}{c} r\in \left(0,1\right). \end{array}$$

If the following formula is satisfied, it is shown in formula (4):

(4) $$\begin{array}{c} q_{i-1}<rq_{i}>r,i>1. \end{array}$$

Then select individual *x*_*i*_; otherwise select individual *x*_1_. It can be seen that, in the roulette algorithm, the third step is more likely to select individuals with high fitness.

The article "Comprehensive Health Evaluation Model of Art Psychotherapy Using Genetic Algorithm" was retracted in 2023. Reasons: unreliable results or conclusions; concerns about the data; concerns about the results or conclusions; concerns about the peer review.

Random traversal sampling algorithm: this algorithm is similar to roulette selection algorithm. The first two steps are also to calculate the individual fitness proportion and fitness distribution. However, in the third step, random traversal sampling adopts the concept of equidistant sampling. Assuming that the number of individuals in the population is *N* and the number of individuals to be selected is *d*, the selection sequence is as shown in formula (5):

(5) $$\begin{array}{c} \left\{r_{1},r_{2},\ldots ,r_{d}\right\}, \end{array}$$

where *r*_1_ is the random number between (0,1/*d*); it is shown in formula (6):

(6) $$\begin{array}{c} r_{j}=r_{j-1}+\frac{1}{d}. \end{array}$$

Tournament selection method: different from the first two, the tournament selection method does not need to calculate the probability distribution function but selects individuals by simulating the way similar to the group competition, which is mainly divided into three steps:

1. Determine the scale of each competition; for example, select 30% of the individuals in the original population to compete.
2. Select the champion (with the highest fitness) among the individuals who meet the number by random sampling.
3. Repeat steps 1 and 2 until a sufficient number of individuals are selected.

Crossover refers to the process of hybridization of parent individuals to produce offspring, which is divided into single point hybridization and multipoint hybridization, as shown in Figure 7.

### 3.3. Clustering Algorithm

#### 3.3.1. Algorithm Process

Clustering technology, also known as cluster analysis, is a technology to analyze the data according to the correlation between the data itself in the absence of prior knowledge. Therefore, clustering is an important part of unsupervised learning, and it is also widely used in pattern recognition, machine learning, and other fields [13].

In cluster analysis, there are two cases—a single data belongs to and only belongs to one category or may belong to multiple categories, corresponding to hard clustering and fuzzy clustering, respectively. In the hard clustering model, the clustering results are shown in formula (7):

(7) $$\begin{array}{c} U=\left[\begin{array}{cccc} u_{11} & u_{12} & \ldots & u_{1n}\\ u_{21} & u_{22} & \ldots & u_{2n}\\ \ldots & \ldots & \ldots & \ldots \\ u_{k1} & u_{k2} & \ldots & u_{kn} \end{array}\right], \end{array}$$

where *U* is the *k* × *n* matrix, where *k* is the number of clusters, *n* is the number of samples, and *u*_*ij*_ indicates whether sample *i* belongs to cluster *j*, which satisfies the following formula, as shown in formula (8):

(8) $$\begin{array}{c} u_{ij}\in \left\{0,1\right\},1\leq j\leq k,1\leq i\leq n. \end{array}$$

In hard clustering, sample *i* either belongs to cluster *j* or does not belong to cluster *j*, and there is no value between 0 and 1. In fuzzy clustering, the formula should be modified as shown in formula (9):

(9) $$\begin{array}{c} u_{ij}\in \left[0,1\right],1\leq j\leq k,1\leq i\leq n. \end{array}$$

In the two different clustering methods, *u*_*ij*_ is also constrained by formulas (10) and (11):

(10) $$\begin{array}{c} \sum_{j=1}^{k}u_{ij}=1,1\leq i\leq n, \end{array}$$

(11) $$\begin{array}{c} \sum_{i=1}^{n}u_{ij}>0,1\leq j\leq k. \end{array}$$

In fuzzy clustering, the sum of distribution probability of samples in all clusters is 0. Formula (11) imposes a basic constraint on the cluster capacity; that is, any existing cluster has at least one sample that belongs or has a probability of belonging to it; otherwise the cluster does not exist [14].

The article "Comprehensive Health Evaluation Model of Art Psychotherapy Using Genetic Algorithm" was retracted in 2023. Reasons: unreliable results or conclusions; concerns about the data; concerns about the results or conclusions; concerns about the peer review.

#### 3.3.2. Algorithm Evaluation Index

The following is a brief introduction to these evaluation indicators: CA: judge whether all samples in the cluster are classified into appropriate clusters by giving a label, and evaluate the clustering effect by statistical accuracy. The calculation is shown in formula (12):

(12) $$\begin{array}{c} CA=\sum_{i=1}^{K}\frac{\max\left(C_{i}|L_{i}\right)}{\left|\Omega \right|}. \end{array}$$

RI and ARI: given the sample label, all point pairs can form four indicators, the same label but belonging to different clusters, the same label and the same cluster, the same cluster of different labels, and different clusters of different labels, as shown in Table 1.
Then the RAND coefficient is calculated with formula (13):
  (13) $$\begin{array}{c} RI=\frac{a+d}{a+b+c+d}. \end{array}$$
In the case of random, the ARI value is close to 0. With the improvement of clustering index, the ARI value is closer to 1. Its calculation method is shown in formula (14):
  (14) $$\begin{array}{c} \text{ARI}=\frac{RI-E\left[RI\right]}{\max\left(RI\right)-E\left[RI\right]}. \end{array}$$
The value range of ARI becomes [−1, 1]. The larger the value, the closer the clustering effect to the real data distribution.
NMI: mutual information (MI) is a concept in information theory, which is mainly used to evaluate the correlation between the distribution of two random variables. There are two random variables *X*, *Y*, *p*(*x*) is the edge distribution of *x*, *p*(*y*) is the edge distribution of *y*, and *p*(*x*, *y*) is its joint distribution; then MI is calculated as formula (15):
  (15) $$\begin{array}{c} MI\left(X,Y\right)=\sum_{x}\sum_{y}p\left(x,y\right)\log\frac{p\left(x,y\right)}{p\left(x\right)p\left(y\right)}. \end{array}$$
Standardized mutual information (NMI) is also called normalized mutual information; that is, standardize the value of mutual information to between [0, 1] through the standardization method, as shown in formula (16):
  (16) $$\begin{array}{c} \text{NMI}\left(X,Y\right)=2\frac{MI\left(X,Y\right)}{H\left(X\right)+H\left(Y\right)}, \end{array}$$
where *H*(·) represents the information entropy of random variables, and the calculation is shown in formula (17):
  (17) $$\begin{array}{c} H\left(X\right)=\sum_{k\in S}p\left(x\right)\log_{2}p\left(x\right). \end{array}$$
Through the above formula, the mutual information between two random variables is normalized to [0, 1]. At the same time, NMI can also correct the bias of MI for more variables.
CP and SP: compactness CP refers to the average distance from each point in the cluster to the cluster center; that is, the smaller the CP value, indicating that the closer the distance within the cluster in the clustering model, the smaller the CP value in theory, the better. The tightness calculation can be calculated by formulas (18) and (19).
  (18) $$\begin{array}{c} CP=\sum_{i=1}^{k}CP_{i}, \end{array}$$
  (19) $$\begin{array}{c} CP_{i}={\left(\frac{1}{\left|C_{i}\right|}\sum_{k\in C_{i}}d^{p}\left(x,c_{i}\right)\right)}^{\left(1/p\right)}. \end{array}$$
DBI index: due to the limitations of CP and SP, it is easy to fall into the local optimal solution when using CP or SP alone to evaluate the clustering model, while DBI balances the two and defines the performance of the clustering model on its basis. The calculation method can be determined by formula (20):
  (20) $$\begin{array}{c} \text{DBI}=\frac{1}{k}\sum_{i=1}^{k}\max_{j\neq i}\left(\frac{CP_{i}+CP_{j}}{{\left\|c_{i}-c_{j}\right\|}_{2}}\right). \end{array}$$
Here is the DBI index description of Euclidean distance. From the definition of DBI, we can see that it takes into account the benefits of CP and SP for the quality evaluation of clustering model. The smaller the DBI value in application, the better.

The article "Comprehensive Health Evaluation Model of Art Psychotherapy Using Genetic Algorithm" was retracted in 2023. Reasons: unreliable results or conclusions; concerns about the data; concerns about the results or conclusions; concerns about the peer review.

## 4. Research on Comprehensive Health Evaluation of Art Psychotherapy

### 4.1. Research Assumptions

The purpose of this study is to compare the experimental effects through quantitative analysis. In the research, mainly guided by the viewpoint of “post-modern experiential art creation,” the intervention group and control group were designed, and the pretest was conducted for group A and group B to ensure the equality of grouping. SPAT group psychological counseling was carried out. After the intervention, the experimental effects of the following aspects were analyzed and compared to explore its internal mechanism [15].

According to the above specific research purposes, the overall research assumptions of the intervention results in the second part of the study are as follows:

  Experimental preconditions: equal histochemical design Pre A = Pre B.
  Expected results of the experiment: paired samples of pretest and posttest in the same group: *t*-test: Post A > Pre A.
  Analysis of variance of posttest comparison of differences between different groups: Post A > Post B.

The specific meanings of the general assumptions are described as follows:

  Hypothesis a: compared with before and after intervention group A, spat group counseling (intervention group A) has significant differences in six aspects: self-harmony, depression, Eysenck personality type, social avoidance and anxiety, life orientation, optimism, and trait coping style [16].
  Hypothesis AB: compared with control group B, spat group counseling has significant differences in six aspects: self-harmony, depression, Eysenck personality type, social avoidance and anxiety, life orientation, optimism, and trait coping style [17].

### 4.2. Implementation Process

The research object of this study is college students. Due to the particularity of the course, after consultation and discussion with relevant teachers and departments before the course, it is possible to implement a unique teaching form of comprehensive painting therapy in a college students' mental health course. The educational intervention of spat curriculum in this study was undertaken by an associate professor of psychology and one of the authors of this paper. The professor has 20 years of teaching experience in psychology. The author is a graduate student majoring in psychology and obtained the qualification certificate of national second-class psychological consultant and secondary vocational teacher. The author is responsible for preparing all the art media required for the course before class. In addition to reading a large number of relevant literature before the course, the interveners also discussed the spat course education plan in detail to ensure the quality of course education [18].

The course site is a fixed large classroom to meet the needs of activities in the course. The selection of specific art media, evaluation tools, and data processing are basically the same as the group counseling part of the second research. It should be noted that the love attitude scale (LAS) used in this study has good structural validity through confirmatory factor analysis. There are 22 items in 6 subscales, and the reliability of each subscale is between 0.706 and 0.818. The concept of love composed of six love styles: romance, game, companion, reality, possession, and dedication also exists among college students in mainland China. The view of love is a multidimensional psychological value. The initially formed love attitude scale can be used as a tool to evaluate the tendency of college students' view of love [19].

The article "Comprehensive Health Evaluation Model of Art Psychotherapy Using Genetic Algorithm" was retracted in 2023. Reasons: unreliable results or conclusions; concerns about the data; concerns about the results or conclusions; concerns about the peer review.

Comprehensive painting art therapy is committed to the unified and coordinated development of students' cognition, emotion, behavior, and personality as a whole. Therefore, different art experience activities such as painting are designed from different levels, and the curriculum education implementation plan is finally determined in combination with the basic teaching content of mental health curriculum [20]. The number of students in this course is 116, collectively known as the intervention group. There are ten courses, one hour and 30 minutes each time. See Table 2 for the specific contents of the curriculum education program.

Comprehensive painting art therapy is committed to the unified and coordinated development of the three levels of cognition, emotion, behavior, and personality of group members. Therefore, different painting and other art experience activities are designed from different levels. At the same time, the group counseling activity plan of this study is finally determined by referring to the existing painting art treatment group plans at home and abroad and under the guidance of professionals [21]. SPAT group psychological counseling activities were carried out for 9 times, once a week, about 2 hours each time. The control group did not intervene. See Table 3 for the specific contents of the activity plan.

The measurement part of the questionnaire is the reevaluation of the psychological scale. Fill in the self-compiled feedback form of group counseling effect, and then give full feedback and discussion between the instructor and members. Finally, the team farewell activity is called “big reunion.” The purpose is to bid farewell to the group in a warm, sweet, and cohesive situation, go to life, and leave a beautiful and unforgettable memory.

### 4.3. Research Results and Discussion

#### 4.3.1. Comparison of Pretest Results of Psychological Measurement between SPAT Group Psychological Counseling Intervention Group and Control Group

Before spat group counseling, the intervention group and the control group were measured with the professional psychological scale. The analysis of variance showed that there was no significant difference between the intervention group and the control group in these aspects. The specific test results on different scales are shown in Table 4.

The article "Comprehensive Health Evaluation Model of Art Psychotherapy Using Genetic Algorithm" was retracted in 2023. Reasons: unreliable results or conclusions; concerns about the data; concerns about the results or conclusions; concerns about the peer review.

#### 4.3.2. The Influence of Educational Intervention of SPAT Course on the Types of Love Attitude

In order to investigate whether there are statistically significant changes in students' love attitude before and after the educational intervention of spat course, the *t*-test of paired samples of “pretest and posttest” is carried out. The results are shown in Table 5.

It can be found from the data in the table that, before and after the experiment, there is a significant difference in the peer love factor in the pretest and posttest results of the intervention group (*P* < 0.05), and there is no significant difference in other factors. There was no significant difference in other factors. This shows that spat curriculum intervention can enhance the tendency of “peer love” and has a positive effect on improving the types of love attitudes of college students. The ternary theory of love holds that love should have three core points: intimacy, passion, and commitment. “Peer love” is the love for intimate partners formed by the combination of intimacy and commitment. This kind of love is characterized by mutual respect and trust between the two sides. What people experience is more a sense of trust and dependence on each other. This type of love will be concentrated in a long and happy marriage. Although the passion is gone, common ideals, common interests, common values, tolerance, and habits can better maintain good feelings. Therefore, more guidance should be given to college students.

#### 4.3.3. Influence of Educational Intervention of SPAT Course on Eysenck's Personality Type Characteristics

In order to investigate whether there are statistically significant changes in the factors of students' Eysenck personality type before and after the educational intervention of SPAT course, the *t*-test of paired samples of “pretest-posttest” is carried out. The results are shown in Table 6.

It can be found from the data in the table that, before and after the experiment, there is an extremely significant difference in EPQ extraversion factor in the pretest and posttest results of the intervention group (*P* < 0.01), and there is no significant difference in other factors. This shows that spat curriculum intervention can significantly improve the extraversion of college students' personality types. The reason may be that the curriculum education improves the openness of members, stimulates their internal spontaneity and initiative, and is willing to show more characteristics such as good communication, enthusiasm, and impulse. Fang Shuren depicted in the curriculum intervention is a specific image and a psychological “self-sufficiency,” resulting in no significant change before and after the educational intervention LOT-R. The comparison results before and after the educational intervention LOT-R are shown in Table 7.

The article "Comprehensive Health Evaluation Model of Art Psychotherapy Using Genetic Algorithm" was retracted in 2023. Reasons: unreliable results or conclusions; concerns about the data; concerns about the results or conclusions; concerns about the peer review.

#### 4.3.4. The Influence of Educational Intervention in SPAT Curriculum on Trait Coping Style

In order to investigate whether there are statistically significant changes in students' trait coping styles before and after the educational intervention of spat course, a paired sample *t*-test of “pretest and posttest” was carried out. The results are shown in Table 8.

It can be found from the data in the table that there is no significant difference between the pretest and posttest results of the intervention group in the negative and positive factors of trait coping style before and after the experiment. The reason may be that the students participating in the curriculum intervention do not have coping style problems, and there is no significant change before and after.

## 5. Conclusion

From the overall results of this study, compared with the control group, spat group psychological counseling significantly enhances college students' self-flexibility, improves the degree of self-harmony, reduces college students' social avoidance tendency, improves college students' extraversion of personality types, has a more positive effect on reducing personality concealment, and can improve college students' optimistic attitude. The positive coping style factor increased, and the scores of other depressive tendencies, neuroticism factors, negative coping styles, and social anxiety factors decreased, which is in line with the initial assumption of this study. The specific research conclusions are as follows.

In the rehearsal group discussion, there was a difference in personal transformation between this group (sampan) and other groups before and after the experiment (*P* < 0.05). There was no significant difference in group B before and after the experiment (*P* > 0.05). After the experiment, there was a significant difference in individual stereotype types between the affected group and the control group (*P* < 0.05), and there was no statistical difference between the other groups (*P* > 0.05).

In the group discussion of art design improvement, there was a significant difference in EPQ concealment (*P* < 0.01) and a significant difference in EPQ extroversion factor (*P* < 0.05) before and after the experiment, but there was no significant difference in the control panel. After the experiment, the difference in EPQ extroversion between the control group and the control group was statistically significant (*P* < 0.05).

The article "Comprehensive Health Evaluation Model of Art Psychotherapy Using Genetic Algorithm" was retracted in 2023. Reasons: unreliable results or conclusions; concerns about the data; concerns about the results or conclusions; concerns about the peer review.

In the group discussion of art deco, there was a significant difference between the groups of avoidance before and after the experiment (*P* < 0.05), and there was no significant difference with other groups. After the experiment, there was a significant difference in the total stress score between the control group and the control group (*P* < 0.05).

In the art deco group discussion, the LOT-R life orientation total score listed in the group was significantly different before and after the experiment (*P* < 0.05), but there was no significant difference in the control group. After the experiment, there was a statistically significant difference in the total score of life direction between the affected group and the control group (*P* < 0.01).

In the group discussion of decorative art design, the adverse effects of TCSQ on the intervention process were significantly different in each group before and after the experiment (*P* < 0.05), but there was no significant difference in the control group. After the experiment, there was no significant difference between the intervention group and the control group in both adverse and positive performance.

With all the benefits of this study, the spat data reported effects on improving college students' romantic behaviors, increasing college students' extroversion, reducing underlying behaviors more effectively, and lowering student relationships and stress. Other factors did not change significantly, but scores increased on positive thinking for good solution quality and positive behavior and increased on other stressors, mental disorders, neurotic factors, and poor resolution, consistent with the original theory. The main points of the special research are as follows:

In the research on the effect of layered art, the point-to-point interaction before and after the experiment was significantly different (*P* < 0.05) and different from others (*P* > 0.05).

In the fine-grained visual art effect research, the EPQ extroversion of each group before and after the experiment was significantly different (*P* < 0.01). There were no significant changes in other factors (*P* < 0.05).

In the study of the effect of art on visual arts, there was no significant change in the composite score of stress and depression in the affected group before and after the study (*P* < 0.05).

In the impact study of medical art presentation, there were significant differences between the pre- and postintervention groups in avoiding social and community stress (*P* < 0.05), and there was a significant difference in avoiding social and community stress (*P* < 0.05) and the total score of grief (*P* < 0.01).

The article "Comprehensive Health Evaluation Model of Art Psychotherapy Using Genetic Algorithm" was retracted in 2023. Reasons: unreliable results or conclusions; concerns about the data; concerns about the results or conclusions; concerns about the peer review.

In the study of the effect of visual arts correction, there was no significant difference in the total score of the LOT-R vital indicator measure between the affected groups before and after the test (*P* > 0.05).

## Figures and Tables

**Figure 1:** Comprehensive evaluation model of artistic psychotherapy health based on genetic algorithm.

**Figure 2:** Feature selection process.

**Figure 3:** Filter feature selection process.

**Figure 4:** Wrapper feature selection process.

**Figure 5:** Principle of genetic algorithm.

**Figure 6:** Coding of a gene.

**Figure 7:** Two hybridization methods.

**Table 1:** Corresponding table of cluster labels.

	Homocluster	Different clusters	Total
Same label	a	b	a + b
Different labels	c	d	c + d
Total	a + c	b + d	a + b + c + d

**Table 2:** Implementation plan of SPAT mental health course.

Course time	Course unit topics	Course implementation process and method	Remarks: art media
1 March 1, 2010	Purpose of family formation: to understand the course form, eliminate the strangeness among members, understand each other, and form a small family	(1) Course introduction: introduce the course content, form, and teaching methods	A4 sketch paper, Hb pencil, eraser, etc.
	Establish reasonable coping styles before, after, or after falling in love	(2) The first test of psychological scale is the pretest	Zhi, glue, scissors, self-brought pictures, and photos related to love, etc.
		(3) Warm-up activities: use the Gestalt grouping method to group according to age, zodiac, and exchange personality characteristics with each other	
		(4) Group grouping “simulated family”: divided into 10 small families, with more than 11 people in each group. Each group selects two principal and deputy parents to be responsible for management and gives a sentence of “who is (she),” and finally shares it	
		(5) Situational drama activities: the performance of “the development process of love emotion” in situational drama, that is, acquaintance, development, conflict, redevelopment, and decision, who is most able to think about their own pursuit and ideas, emotional needs, and how to actively guide	

9 May 10, 2010	Emotional integration purpose: to integrate friendship, family affection, and love emotion from the level of knowing and doing	(1) Introduction to the course: the explanation of love sentiment, that is, sense of reason, aesthetics, and morality	24 color watercolor pens, oil painting stick, color pencil, A4 sketch paper, Hb pencil, eraser, etc.
		(2) Emotional test and case discussion and explanation	
		(3) Painting and story analysis: “future life—a better tomorrow” nine-division painting and story sharing, according to the operation steps of the nine-division integration painting method	
		(4) Viewing of audiovisual materials: emotion and marital emotion	

10 May 17, 2010	The purpose of personality integration: members share deeply, integrate the curriculum harvest, and integrate into personality	(1) Course introduction: course summary	Watercolor pen, oil painting stick, watercolor pigment, rice paper, A4 sketch paper, pencil, eraser, etc.
		(2) Personal painting: “a growing tree of life” and sharing	
		(3) Group painting: “emotional garden,” small family as a group, using large rice paper	
		(4) Explore the future career blueprint, discuss, and share	
		(5) After the second test of the psychological scale, the students bid farewell to each other	

The article "Comprehensive Health Evaluation Model of Art Psychotherapy Using Genetic Algorithm" was retracted in 2023. Reasons: unreliable results or conclusions; concerns about the data; concerns about the results or conclusions; concerns about the peer review.

**Table 3:** SPAT group psychological counseling program.

Activity name	Activity objectives	Process and method	Art media
(1) A new family 2010.03.04	(1) Clarify the objectives of the group and the formation of the group	(1) Introduction and discussion on the content and form of group activities (20 minutes)	Watercolor pen, color pencil, oil painting stick, color small cardboard; psychological scale and informed consent
	(2) Be familiar with team members and art media	(2) Psychological scale measurement and signing informed consent (20 minutes)	
	(3) Build trust and warm group atmosphere	(3) Warm-up activities—social measurement and body bumper car (20 minutes)	
		(4) Set up three small families to discuss and display “family name,” “family number,” “family song,” and “family dance” (25 minutes)	
		(5) Nine-cell emotional painting (20 minutes)	
		(6) End sharing (15 minutes)	

(2) Who am I 2010.03.11	(1) Emphasize group commitment and enhance group motivation	(1) Group dynamic reconstruction (15 minutes)	2B pencil, eraser, A4 sketch paper: oil paint, rice paper, brush, platter;
	(2) Improve self-awareness	(2) Self-portrait painting (30 minutes)	
		(3) Music image painting (30 minutes)	

**Table 4:** Results of pretest ANOVA of psychological scale in intervention group and control group.

Scale and its factor name	Group	*N*	Mean	SD	Variance homogeneity test			Analysis of variance results
					Levene statistics	Sig. (*P* value)	*F* value	*P*
Disharmony factors of SCCS self and experience	Intervention group A	15	41.470	6.543	2.430	0.130	1.802	0.190
SCCS self-spirit	Control group B	15	46.070	10.879				
	Intervention group A	15	21.730	3.918				

**Table 5:** *T*-test results before and after spat curriculum education intervention love attitude scale.

Paired comparison of pretest and posttest differences			*T*-test results	
Scale and factor name	Mean	SD	*T* value	*P*
Romantic love	0.257	2.557	1.030	0.305
Game love	−0.124	3.021	−0.420	0.675
Companion love	0.705	3.079	2.346	0.021^*∗*^
Possessive love	−0.114	2.569	−0.456	0.650
Realistic love	−0.105	2.382	−0.451	0.653
Give love	−0.057	2.541	−0.230	0.818

^*∗*^ *P* < 0.05, ^*∗∗*^*P* < 0.01.

The article "Comprehensive Health Evaluation Model of Art Psychotherapy Using Genetic Algorithm" was retracted in 2023. Reasons: unreliable results or conclusions; concerns about the data; concerns about the results or conclusions; concerns about the peer review.

**Table 6:** Results of *t*-test before and after the short EPQ scale of educational intervention in SPAT course.

Paired comparison of pretest and posttest differences			*T*-test results	
Scale and factor name	Mean	SD	*T* value	*P*
EPQ psychoticism factor	−0.123	1.357	−0.935	0.352
EPQ extraversion factor	−0.686	2.105	−3.339	0.001^*∗∗*^
EPQ neuroticism factor	−0.019	2.780	−0.070	0.944
EPQ masking factor	0.076	1.895	0.412	0.681

^*∗*^stands for *P* < 0.05, ^*∗∗*^*P* < 0.01.

**Table 7:** *T*-test results before and after LOT-R of educational intervention in SPAT course.

Paired comparison of pretest and posttest differences			*T*-test results	
Scale and factor name	Mean	SD	*T* value	*P*
Total score of LOT-R life orientation scale	−0.029	3.712	−0.079	0.937

^*∗*^ *P* < 0.05, ^*∗∗*^*P* < 0.01.

**Table 8:** *T*-test results before and after TCSQ of educational intervention in spat course.

Paired comparison of pretest and posttest differences			*T*-test results	
Scale and factor name	Mean	SD	*T* value	*P*
TCSQ negative coping style factor	−0.038	5.932	−0.066	0.948
TCSQ positive coping style factor	−0.419	6.978	−0.615	0.540

^*∗*^ *P* < 0.05, ^*∗∗*^*P* < 0.01).

## Data Availability

The labeled data set used to support the findings of this study is available from the corresponding author upon request.
